# Expression of Hypersensitive Troponin I and Soluble ST2 in Acute Organophosphorus Pesticide Poisoning

**DOI:** 10.1155/2022/1427231

**Published:** 2022-01-27

**Authors:** Xiaoting Liu, Lei Wang, Jing Chen, Hongna Qi, Guoying Ma, Weizhan Wang

**Affiliations:** Department of Emergency, Hengshui People's Hospital, Hengshui, Hebei 053000, China

## Abstract

The role of soluble growth stimulating gene 2 protein and highly sensitive cardiac troponin in the diagnosis of early myocardial injury caused by acute organophosphorus pesticide poisoning was studied. 171 inpatients with AOPP were divided into three experimental groups according to their mild, moderate, and severe conditions. 20 healthy people were selected as the control group. The levels of cTnI, HS-CTNI, NT proBNP, and ST2 were measured at the 4th and 12th hours after the experiment. The measured data were expressed by mean standard deviation. The independent sample *t*-test was used for the detection between the two groups, and one-way ANOVA was used for the analysis and comparison between multiple groups. The relevant data were analyzed by Spearman correlation test (*P* < 0.05). The levels of cTnI and HS cTnI in the experimental group increased with the extension of time and the deepening of poisoning degree; four hours after admission, ST2 and NT proBNP water in the control group and the experimental group increased significantly on average. According to the analysis of the data, there was a positive correlation between HS TnI and ST2 in patients with AOPP (*r* = 0.938, *P* < 0.001, *r* = 0.827, *P* < 0.001). The more serious the disease, the higher the concentrations of HS TnI and ST2, and the more serious the myocardial injury.

## 1. Introduction

Our country is agricultural country, many poisoning patients, including acute organophosphorus pesticide poisoning (acute organophosphoruspesticide poisoning, AOPP) of emergency poisoning disease first [1], the onset of fierce, rapid progress, and high mortality [2]. The toxicity will cause multiple organ function damage, and the myocardial cell damage is the most serious. The present study shows that hypersensitive troponin I (HS-TNI) can indicate early myocardial injury better than conventional troponin [3]. Soluble growth stimulation expression gene 2 protein (sST2) belongs to interleukin-1 receptor, which is a serum protein secreted by myocardial cells and myocardial fibroblasts when stimulated, indicating myocardial necrosis [4]. The purpose is to study the relationship between HS-TNI and sST2 and the myocardial injury induced by AOPP.

## 2. Data and Methods

### 2.1. General Clinical Data

171 AOPP patients treated in the emergency department of Hengshui people's Hospital from August 2016 to October 2019 were selected for the experiment. Among them, all patients met the AOPP diagnostic criteria in the eighth edition of internal medicine [5]. The poisoning route was oral, 50-200 ml drug, and the poisoning time was within 2 h. Among AOPP patients, there were 67 cases of methamidophos poisoning, 37 cases of parathion poisoning, 47 cases of dimethylamine poisoning, and 20 cases of dichlorvos poisoning. There were 78 males and 93 females, of which 171 were aged from 18 to 55 years, with an average age of 43.11 ± 2.15 years.

### 2.2. Diagnosis, Treatment, and Grouping after Admission

171 patients with AOPP were hospitalized after routine treatment due to acute organophosphorus pesticide poisoning. According to the eighth edition of internal medicine, 171 patients with AOPP were divided into three experimental groups according to the dose of pesticides ingested by mistake and the harm degree of different pesticide components, including 46 cases in the mild group, 56 cases in the moderate group, and 69 cases in the severe group. After treatment, all patients improved without death. Twenty healthy people without any disease were selected as the control group, including 10 males and 10 females, aged from 30 to 55 years, with an average of 43.15 ± 3.80 years. There was no significant difference between the two experimental groups in other aspects, *P* > 0.05.

### 2.3. Detection and Observation Indicators

In this experiment, the automatic detection analyzer of heart reader is selected to detect cTnI (0-0.5 ng/ml), HS cTnI (0-0.08 ng/ml), and NT proBNP (0-250). This instrument is an existing common detection instrument in the hospital. At the same time, 5 ml blood samples were collected at the speed of 3000r/min and centrifuged for 10 min to separate the serum. Soluble growth stimulating gene 2 (sst2) protein (< 35 ng/ml) was detected by enzyme-linked immunosorbent assay (ELISA). The toolkit was developed by C & amp, provided by company D. The research scheme of this subject has been approved by the hospital ethics committee, and the patients participating in the experiment have also received the support and consent of their families. The symptoms and ECG of poisoning patients were observed.

### 2.4. Statistical Methods

The data were analyzed by SPSS 21 software. The independent samples were normally distributed. The experimental data are measured in the way of average standard deviation, the pairwise comparison between the data is checked by the *t*-test method of independent samples, and the test of multiple groups of data is checked and compared by the way of univariate. Count data 2 × 2 table comparison between groups using *X*^2^ test; Spearman correlation coefficient test is used for correlation analysis between data. *P* value represents the test level. If *P* < 0.05 is measured, it indicates that there is a statistical difference. The *F* value of ANOVA was used to evaluate the difference between groups. The greater the *F* value, the better the significance as shown in Figure 1.

## 3. Experimental Process

### 3.1. Comparison of General Clinical Data of Patients in AOPP Poisoning Groups

There is no obvious difference in clinical data between AOPP patients with different degrees of poisoning, such as gender, age, weight, and time to visit the doctor for poisoning (*P* > 0.05). In terms of toxic dose, there was significant statistical significance among the groups (*P* < 0.05). See Table 1.

### 3.2. Dynamic Comparison of cTnI and HS-CTNI in Each Group of AOPP Patients

The levels of serum cTnI and HS cTnI in AOPP patients at different times were compared, which were divided into 1 hour, 4 hours, and 12 hours. See Table 2 for specific conditions of experimental measured data:

The serum HS cTnI level of AOPP patients with different 1-hour poisoning degrees was higher than that of the control group (healthy people). Compared with the mild group, the poisoning degree in the severe group was higher than that in the mild group, but there was no significant difference in cTnI level between the two groups (*P* > 0.05), and there was significant difference between the two groups (*P* < 0.05). It was found that the levels of cTnI and HS cTnI in the experimental group increased with the increase of time and poisoning degree. The test results within 12 hours were significantly higher than those within 4 hours. There was significant difference between severe group and mild group (*P* < 0.05), indicating that the measurement data were statistically significant as shown in Figure 2.

### 3.3. Comparison of NT-probNP and sST2 in Each Group of AOPP Patients

According to the serum NT proBNP and ST2 levels of AOPP patients at different times, they were divided into 1 hour, 4 hours, and 12 hours. The comparison of NT pronp and ST2 concentrations in patients *d* with different degrees of poisoning is shown in Table 3.

One hour after admission, the level of ST2 in the experimental group was higher than that in the control group. In the experimental group, ST2 in the severe group was higher than that in the mild group and moderate group, and the measured data between groups were statistically significant (*P* < 0.05). At 4 and 12 hours after admission, the results showed that ST2 in the experimental group and the control group increased, and the increase was most obvious in the severe group. The SST measured at 212 hours in each group was significantly higher than that measured at 4 hours. There was significant statistical significance in the comparison of measurement data among groups. At 1 h after admission, NT proBNP in each group was within the normal range. At 4H and 12 h after admission, NT proBNP gradually increased with time, and the severe group was significantly higher than the control group, which confirmed that NT proBNP could evaluate the severity of AOPP myocardial injury. The more severe the myocardial injury, the higher the level of ntprobnp. With the aggravation of AOPP poisoning, the level of NT proBNP increased gradually. The comparison between ST2 and ST2 was statistically significant (*P* < 0.05).

### 3.4. Correlation Analysis of HS-TNI and sST2 with AOPP

According to the analysis of the obtained data, there is a positive correlation between Hs-TNI and sST2 in AOPP patients (*R* = 0.938, *P* < 0.001, *R* = 0.827, *P* < 0.001). The more serious the patient's condition, the higher the concentration of Hs-TNI and sST2, and the more severe the myocardial injury.

Through the data analysis of the research results, it can be found that the ST2 of the moderate and severe groups in the experimental group is higher than that of the control group and also higher than that of the mild and moderate groups in the experimental group. Compared with the control group, the difference was statistically significant (*P* < 0.05). In addition, the level of ST2 in the experimental group and the control group increased at 4 and 12 hours, especially in the severe group. ST2 increased significantly at 12 hours after admission compared with 4 hours after admission (*P* < 0.05).

## 4. Discussion

The mechanism of myocardial injury after AOPP poisoning is as follows: (1) toxin directly damages cardiomyocytes [6]; (2) the accumulation of acetylcholine leads to the abnormal destruction of ion channels and the inhibition of cardiac conduction system [7]; (3) a series of inflammatory reactions were induced after poisoning, and the inflammatory response conduction of cardiomyocytes was inhibited [8]; (4) vomiting and gastric lavage during treatment resulted in electrolyte disorder and increased blood concentration and blood viscosity [9]; and (5) poisoning causes sympathetic nerve excitation. Anticholinergic drug treatment leads to increased heart rate and myocardial oxygen consumption, aggravating cell ischemia and hypoxia, leading to coronary artery spasm, decreased myocardial contractility, malignant arrhythmia, and even sudden cardiac death. Early detection, early diagnosis, and early treatment should be taken for AOPP poisoning [10], which will help to shorten the average length of hospital stay, reduce hospitalization expenses, and reduce mortality.

When the heart is damaged due to AOPP poisoning, a large amount of cTnI is released into the blood, which can be detected 3-6 hours after the onset and reach the peak at 18-24 hours, and the blood concentration can be maintained for 6-10 days [11]. However, the level of cTnI in blood circulation is often low; so, there may be a risk of misdiagnosis and missed diagnosis [12]. With the wide application of HS cTnI (high-sensitivity troponin I) detection, its hypersensitivity and lower concentration threshold can detect more myocardial necrosis. Relevant reports found that [13] the level of serum hs-ctni increased within 3 hours after myocardial injury. For the symptoms of patients with suspected weak myocardial injury, HS cTnI can be detected to improve the detection rate and can be combined with other myocardial markers; compared with cTnI detection time, the concentration of HS cTnI increased significantly, which can better carry out clinical evaluation and guide treatment strategies. The results of this study show that hs-ctni plays an important role in the early diagnosis of myocardial injury in patients with AOPP.

In addition, as a new biomarker, sst2 can reflect inflammation, fibrosis, and myocardial tension at the same time and can predict the occurrence of adverse cardiovascular events [14, 15]. ST2 increased 2-4 hours after onset, peaked at 6-17 hours, and gradually decreased 1 week after onset, which was not related to NT proBNP [16, 17]. In the case of myocardial ischemia and hypoxia after AOPP poisoning, cardiomyocyte injury and necrosis lead to the activation of local monocyte macrophage system, and the proinflammatory cytokines in the injured tissue activate the secretion of ST2 by adjacent cardiomyocytes [18].

Myocardial ischemia and hypoxia are important promoters of NT proBNP release [19], which are directly released from damaged or necrotic cardiomyocytes. In addition, myocardial necrosis increases ventricular tension, leads to changes in local ventricular wall tension and load, leads to abnormal ventricular wall motion and decreased cardiac function, and further stimulates the synthesis and secretion of NT proBNP [20]. NT proBNP level is closely related to cardiac function and myocardial ischemia and necrosis. However, it is susceptible to age, renal function, and weight.

According to the above data, the early degree of myocardial injury in patients with AOPP can be identified by detecting the levels of HS cTnI and ST2, so as to evaluate the degree of myocardial injury more objectively. Both were also positively correlated with the severity of AOPP. It is suggested that hs-tni combined with ST2 can better evaluate the early myocardial injury after poisoning. The degree of myocardial injury can be seen from the concentration of hs-tni. The higher the concentration, the more serious the injury. The decrease of serum cholinesterase cannot fully reflect the degree of organophosphorus pesticide poisoning, let alone evaluate the situation of myocardial injury.

## 5. Conclusion

This paper studied the diagnosis of soluble growth stimulating gene 2 protein ST2 and highly sensitive cardiac troponin IHS cTnI for early myocardial injury caused by acute organophosphorus pesticide poisoning. 171 inpatients with AOPP were divided into three groups (experimental group) and 20 healthy people (control group). The levels of cTnI and HS-CTNI in the experimental group increased with the extension of time and the deepening of poisoning degree; ST2 and NT proBNP water increased significantly on average. By detecting the levels of HS-CTNI and ST2, the degree of early myocardial injury in patients with AOPP can be determined, so as to evaluate the degree of myocardial injury more objectively.

To sum up, when the AOPP caused human myocardial injury, we can know and evaluate the degree of human myocardial injury through early detection and detection of HS-CTNI and sST2 levels and timely guidance and adjustment of therapeutic measures, reduce the further deterioration of cardiac function, reduce the disability rate, and improve the long-term prognosis.

## Figures and Tables

**Figure 1:** Correlation between hs-TnI and severity of AOPP.

**Figure 2:** Correlation between sST2 and severity of AOPP.

**Table 1:** Comparison of clinical data of patients with different levels of poisoning ($\bar{x+s}$).

Group	Gender (female)%	Age	Weight	Poisoning diagnosis time	Toxic dose
Mild 46	25 (54.35)	41.43 ± 2.02	65.93 ± 5.11	1.72 ± 0.04	62.76 ± 5.32
Moderate 56	30 (53.57)	40.83 ± 3.49	65.32 ± 6.15	1.68 ± 0.08	93.26 ± 3.66^a^
Severe 69	35 (50.72)	42.05 ± 1.89	66.17 ± 5.96	1.77 ± 0.03	142.74 ± 4.31^a,b^

In contrast to mild, ^a^*P* < 0.05; compared to moderate, ^b^*P* < 0.05.

**Table 2:** Comparison of cTnI and hs-ctni concentration in patients with different degrees of poisoning ($\bar{x+s}$).

Indicators	The control group of 20	Mild 46	Moderate 56	Severe 69	*F*	*P*
cTnI (ng/ml)	0.12 ± 0.04					
1 h after admission		0.32 ± 0.05	0.32 ± 0.03	0.31 ± 0.04	1.923	0.169
4 hours after admission		0.57 ± 0.04	0.72 ± 0.07	1.34 ± 0.06	2.266	0.001
12 hours after admission		0.68 ± 0.04	0.97 ± 0.08	2.86 ± 0.14	1.653	0.001
hs-cTnI (ng/ml)	0.04 ± 0.01					
1 h after admission		0.11 ± 0.02	0.23 ± 0.03	0.35 ± 0.03	3.536	0.001
4 hours after admission		0.22 ± 0.04	0.52 ± 0.05	1.26 ± 0.04	3.968	0.001
12 hours after admission		0.36 ± 0.06	1.34 ± 0.08	4.28 ± 0.11	1.524	0.001

Compared with 1 h after admission, *P* < 0.05; compared with 4 h after admission, *P* < 0.05.

**Table 3:** Comparison of NT-probNP and sST2 concentration in patients with different degrees of poisoning ($\bar{x+s}$).

Indicators	The control group of 20	Mild 46	Moderate 56	Severe 69	*F*	*P*
NT-proBNP (pg/ml)	167.46 ± 27.22					
1 h after admission		168.04 ± 25.51	172.67 ± 22.83	161.40 ± 21.39	4.688	0.101
4 hours after admission		260.34 ± 19.02^1a^	344.09 ± 22.46^12a^	416.85 ± 23.52^123a^	2.341	0.001
12 hours after admission		595.26 ± 21.83^1ab^	693.24 ± 26.56^12ab^	967.14 ± 30.92^123ab^	1.220	0.001
sST2 (ng/ml)	18.13 +/- 1.71					
1 h after admission		37.07 ± 3.29^1^	43.16 ± 8.49^1a^	49.68 ± 9.32^1ab^	9.047	0.001
4 hours after admission		40.89 ± 5.79^12^	46.69 ± 12.02^12a^	52.28 ± 10.08^12ab^	8.820	0.001
12 hours after admission		46.59 ± 5.71^123^	54.51 ± 11.71^123a^	78.49 ± 12.60^123ab^	4.902	0.001

Note: compared with the control group,^1^*P* < 0.05; in contrast to mild,^2^*P* < 0.05; compared to moderate, ^3^*P* < 0.05; compared with 1 h after admission, ^a^*P* < 0.05; compared with 4 h after admission, ^b^*P* < 0.05.

## Data Availability

The data underlying the results presented in the study are available within the manuscript.
